This article has been retracted.

# Selenium-enriched polysaccharides from *Pyracantha fortuneana* (Se-PFPs) inhibit the growth and invasive potential of ovarian cancer cells through inhibiting *β*-catenin signaling

**DOI:** 10.18632/oncotarget.8619

**Published:** 2016-04-06

**Authors:** Qianling Sun, Mengmeng Dong, Zhihui Wang, Changdong Wang, Deqiao Sheng, Zhihong Li, Debin Huang, Chengfu Yuan

**Affiliations:** ^1^ College of Medical Science, China Three Gorges University, Yichang, HuBei 443002, China; ^2^ Renhe Hospital of China Three Gorges University, Yichang, HuBei 443002, China; ^3^ Molecular Medicine & Cancer Research Center, Chongqing Medical University, Chong qing 400016, China; ^4^ Department of Pharmacology, Hubei Institute for Nationalities, Enshi, HuBei 445000, China

**Keywords:** selenium-enriched polysaccharides, ovarian cancer, antitumor activity, GSK-3β, β-catenin

## Abstract

Polysaccharides from medicinal plants exert antitumor activity in many cancers. Our previous study demonstrated that polysaccharides extracted from the selenium-enriched *Pyracantha fortuneana* (Se-PFPs) showed antiproliferative effect in breast cancer cell line. This study aimed to investigate the antitumor effect of Se-PFPs in ovarian cancer cells *in vitro* and *in vivo.* Se-PFPs could decrease cell viability, induce apoptosis, and inhibit migratory and invasive potentials in HEY and SKOV3 cells. These findings are supported by reduced expression of cyclin D1, Bcl-2 and MMP-9, enhanced cleavage of PARP and caspase-3, elevated activity of caspase-3 and caspase-9, and EMT (epithelial to mesenchymal transition) inhibition (elevated expression of E-cadherin and cytokeratin 19, and reduced expression of N-cadherin, vimentin, ZEB1 and ZEB2). Moreover, Se-PFPs inhibited xenografted tumor growth through inhibiting cell proliferation and inducing cell apoptosis. More importantly, Se-PFPs significantly reduced cytoplasmic *β*-catenin particularly nuclear *β*-catenin expression but increased *β*-catenin phosphorylation in a GSK-3β-dependent mechanism. Furthermore, *β*-catenin knockdown exerted similar effects on cell proliferation and invasion as seen in Se-PFPs-treated cells, while *β*-catenin overexpression neutralized the inhibitory effects of Se-PFPs on cell proliferation and invasion. Take together,Se-PFPs exert antitumor activity through inhibiting cell proliferation, migration, invasion and EMT, and inducing cell apoptosis. These effects are achieved by the inhibition of *β*-catenin signaling. Thus Se-PFPs can be used as potential therapeutic agents in the prevention and treatment of ovarian cancer.

## INTRODUCTION

Ovarian cancer (OC) is the most lethal gynecological malignancy with obstinate abilities of invasion and metastasis [1]. Because the early symptoms of OC are too atypical to diagnose, the primary tumor in the majority of OC patients has already been metastasized to other tissues or organs when it was diagnosed [2]. Cytoreductive surgery is a well-accepted standard treatment for primary OC, while in advanced stages of OC, adjuvant platinum/taxane chemotherapy along with treatment of anti-angiogenic agent such as bevacizumab has been extensively applied [3, 4]. Unfortunately, the majority of OC patients who initially present with advanced disease will relapse [5]. Recurrent OCs become more aggressive and resistant to therapies, and patients will ultimately die of this disease with a median overall survival (OS) of approximately 12 months after the development of drug resistance [3, 5]. Increasing evidence demonstrated that chemoresistance is highly associated with acquiring the capacity of epithelial to mesenchymal transition (EMT) in ovarian cancer cells [6]. Moreover, major signaling pathways such as Wnt/β-catenin, TGF-β and Notch are involved in EMT in OC cells [7, 8].

It is well-accepted that complementary or alternative therapies such as herbal or natural products can significantly enhance standard-of-care therapy, prolong progression-free survival (PFS) and improve quality of life in cancer patients [9]. Some Chinese herb extracts such as ginsenoside 20(S)-Rg3 [10], polyphyllin D [9] and β-Elemene [11] have been found to exert anti-tumor activity in OC cells. In recent decades, the polysaccharides from the medicinal plants have significant bioactivities in anti-tumor, antioxidation, anticoagulation, antidiabetes, radioprotection, antivirus, hypolipidemics and immunomodulation [12, 13]. Moreover, medicinal plant polysaccharides are non-toxic and without side effects, which make them suitable for medicinal treatment applications [12].

Selenium (Se) is a micronutrient element with indispensable biological functions and plays an important role in cancer therapy [14, 15]. Consumption of the appropriate dosage of selenium has been found to exhibit multiple beneficial effects on human health such as the prevention of cancer and cardiovascular diseases [16]. In the body, inorganic Se can be transformed into safe and absorbable organic Se by coupling with polysaccharides and proteins [17]. Compared to Se-free polysaccharides, Se-polysaccharides displayed a significantly stronger antioxidant activity *in vivo* and *in vitro* [18]. Recent studies demonstrated that Se-polysaccharides isolated from medicinal plants exert antitumor activity in human breast cancer cells [19] and murine H22 ascitic hepatoma cells and S180 sarcoma cells [20]. In our previous study, we successfully purified Se-enriched polysaccharides from *Pyracantha fortuneana* (Se-PFPs), which consisted of carbohydrate (93.7%), uronic acid (2.1%), and 3.7 μg/g of Se [21]. Moreover, we demonstrated that Se-PFPs could attenuate CCl_4_-induced liver injury in mice [21]. Although the antitumor activity of Se-polysaccharides has been reported in a couple of cancer types [19, 20], the underlying molecular mechanisms have rarely been clarified.

In the present study, therefore, we investigated the antitumor activity of Se-PFPs in OCs using *in vivo* and *in vitro* techniques and underlying molecular mechanisms. Our results demonstrated that Se-PFPs can induce apoptosis and inhibit the proliferative and invasive potentials in HEY and SKOV3 cells by inhibiting β-catenin signaling pathway, suggesting that Se-PFPs are promising medicines for treating or preventing ovarian cancer.

## MATERIALS AND METHODS

### Reagents and cell lines

The extraction and component analysis of Se-PFPs were performed as described previously [21, 22]. Primary antibodies to Bax, Bcl-2, E-cadherin, N-cadherin, Cytokeratin 19, Vimentin, ZEB1, ZEB2, MMP-9, β-catenin, GSK-3β, CyclinD1, phosphorylated GSK-3β, phosphorylated β-catenin, cleaved caspase-3 and PARP were purchased from Santa Cruz Biotechnology (Santa Cruz, CA, USA). α-tubulin and lamin A/C antibodies (cell signaling technology), MG132 was purchased from Sigma. HEY and SKOV3 cells were initially obtained from American Type Culture Collection (ATCC, Manassas, VA, USA) and maintained in RPMI-1640 medium with 10% fetal bovine serum (FBS), 100 units/ml penicillin and 100 μg/ml streptomycin at 37°C under 5% CO_2_.

### MTT assay

Cell viability was measured as previously described [23]. Briefly, HEY and SKOV3 cells (4,000 cells/well) were grown in 96-well plates in triplicates, and treated with 0, 50, 100, 200, 400, 800 and 1000 μg/ml of Se-PFPs for 24 and 48 hrs. The cells were incubated with 0.5 mg/ml MTT for 4 hrs. The absorbance at 570 nm was assayed.

### Apoptosis assay

HEY and SKOV3 cells were treated with 0, 200 and 400 μg/ml of Se-PFPs for 48 hrs. Then the cells were stained with AnnexinV-fluorescein isothiocynate (FITC) and 50 μg/ml propidium iodide for 15 min in the darkness. The apoptotic cells were analyzed immediately using flow cytometry.

### Cell migration and invasion assays

Serum-starved HEY and SKOV3 cells (50,000 cells/well) were added in duplicate to Boyden chambers with polycarbonate membranes (8 μm pore size, 6.5-mm diameter) (Transwell, Corning Life Sciences, Acton, MA) or to Matrigel invasion chambers with polyethylene terephthalate membrane (8 μm pore size, BD Biosciences). The culture medium in top chamber contained 0, 200, and 400 μg/ml Se-PFPs. After 24 hrs migration/invasion towards media containing 10% FBS, cells on top membrane were removed using a cotton swab, while cells on the lower membrane were fixed with methanol and stained with Giemsa solution (Sigma, St. Louis, MO, USA). Ten fields per well were photographed randomly under light microscopy and the mean cell number in each field was counted using Image-pro plus software.

### Wound healing assay

HEY and SKOV3 cells were grown to 100% confluence in 6-well plates. The cell monolayer of each well was scratched to generate a “scratch wound” using a 200-μl pipette tip. Cells were cultured in serum-free medium with 0, 200, and 400 μg/ml of Se-PFPs for 24 hrs. The wound closure was photographed under an inverted microscope (Nikon Ti, Nikon Corp., Tokyo, Japan).

### MMP-9 activity assay

HEY and SKOV3 cells were treated with 0, 200, and 400 μg/ml Se-PFPs for 48 hrs. Cell culture medium was collected. The standards and medium samples were incubated with MMP-9 monoclonal antibody for 2 hrs, then treated with p-aminophenylmercuric acetate for another 2 hrs at 37°C. The fluorogenic substrate was added and incubated for 20 hrs at 37°C in the dark. The plates were measured at 320 nm of excitation wavelength and 405 nm of emission wavelength on a spectrophotometer.

### Construction of lentiviral plasmids and production of lentivirus particles

β-catenin shRNAs and negative control shRNA were successfully cloned into lentiviral pLKO.1 vector and re-named LV-β-catenin shRNA and LV-NC shRNA, respectively. The full-length of β-catenin was successfully cloned into lentiviral pLVX-AcGFP1-N1 vector (LV-β-catenin), while empty vector was named LV-vector. Lentiviruses were produced in HEK-293T cells. Briefly, HEK-293T cells (2×10^6^) were plated in a 10-cm dish. After 24 hrs, the cells were transfected with 4.0 μg of pMD2.G, 4.0 μg of pSPAX2 and 5.0 μg of lentiviral target plasmids by Lipofectamine 2000 (Invitrogen, USA). The medium was replaced at 8 hrs after transfection and cultured for another 24 hrs. Cell culture medium containing lentivirus particles was collected and filtered through a 0.45 μm filter (Millipore, Billerica, MA, USA). The lentivirus particles were used to infect HEY and SKOV3 cells.

### Real-time reverse transcription PCR

The extraction of total RNA and synthesis of cDNA were performed as previously described [24]. SYBR Green Master Mix kit (Qiagen, Hilden, Germany) was used to perform real-time PCR. The amplification was carried out as follows: 50°C for 2 min; 95°C for 10 min; subsequently 40 cycles of 95°C for 15 sec and 60°C for 60 sec. The relative expression of mRNA was calculated by 2^−ΔΔCt^ method, while GAPDH was used as an endogenous control. PCR primers are listed in Supplementary Table S1 in the supplementary materials.

### Western blot

HEY and SKOV3 cells were treated with indicated concentrations of Se-PFPs for 24 or 48 hrs. Protein extraction and concentration measurement were performed as previously described [21]. For the extraction of nuclear proteins, cells were lysed in hypotonic buffer (10 mM HEPES-KOH, 1.5 mM MgCl2, 10 mM KCl, 0.5 mM DTT, 0.2 mM PEFA, pH 7.9, 0.5% NP-40). Cell lysates were centrifuged for 10 s at 16,000 g at 4°C. The supernatants were collected (cytoplasmic extract, Cyto), and the pellets were washed twice with hypotonic buffer, and lysed with high-salt buffer (450 mM NaCl, 1 mM PMSF, 50 mM Tris pH 7.4, 0.2 mM Na3VO4, 5 mM β-glycerophosphate, 20 % glycerol, 2 mM DTT, 1 % NP-40), following incubation for 10 min on an end-over-end rotator at 4°C. Cell lysates were centrifuged for 15 min at 16,000 g at 4°C, and the supernatants were collected (nuclear extract, Nuc). Denatured proteins (50 μg/well) were separated by 8-15% SDS-PAGE and transferred onto polyvinylidene fluoride (PVDF) membrane. After blocking with 5% fat-free milk for 1 hr, the membrane was incubated with primary antibodies diluted at 1:500 or 1:1000 overnight, and then incubated with appropriate secondary antibodies for 1 hr. β-actin was used as the loading control. The antibody-bound proteins were detected using enhanced chemiluminescence (ECL) Super Signal reagent (Pierce, Rockford, USA) and exposed to the X-ray film by autoradiography.

### Animal experiments

BALB/C female nude mice aged 30 days were used in our study. The animal experimental protocols were in accordance with the Ethics Committee Guide of China Three Gorges University. 1×10^6^ HEY cells were subcutaneously injected into the flank of the mice. The mice were randomly assigned into two groups, with eight mice per group. In the meantime, the mice in the treatment group received one gavage of 400 mg/kg/day of Se-PFPs for 28 consecutive days, while the same volume of vehicle (PBS) was given to the control mice. The size of tumor in two groups was measured on days 7, 14, 21 and 28 after injection using a vernier caliper. After the last gavage, the mice in two groups were fasted for 24 hrs, weighed and euthanized using CO_2_ inhalation. The tumors were then excised and weighed. The tumor volume was calculated with the formula: π/6 × length × width^2^ [24].

### Immunohistochemistry

Tumor tissues were fixed in 4% formaldehyde solution, embedded in paraffin, and then cut into 4-mm serial sections. The immunohistochemical experiment was carried out using the commercial ultra sensitive TM SP Kit (Zhongshan Corp., Beijing, China) following the manufacturer's instructions. The sections were stained with Ki-67 antibody (Santa Cruz Biotechnology) at 1:200 dilution and β-catenin antibody (Santa Cruz Biotechnology) at 1:500 dilution. The negative control was carried out by replacing primary antibody with PBS. For TUNEL (TdT-mediated dUTP nick end labeling) staining, after fixation for 10 minutes with 4% formaldehyde, the slides were treated with acetic acid/ethanol (1:2) for 5 minutes, and incubated at 37°C for 1 hour with terminal transferase mixture (0.25U/L terminal transferase, 2.5 mM CoCl_2_, and 2 pmol fluorescein-12-dUTP (Boehringer Mannheim, Indianapolis,IN). The slides were mounted with Vectashield with propidium iodide (Vector Laboratories, Burlingame, CA) and visualized using fluorescence microscopy. The immunohistochemical staining was scored as previously described [24].

### Statistical analysis

The data from three independent experiments were presented as mean ± standard deviation (SD). Statistical analyses were performed using Student's *t*-test or one-way analysis of variance (ANOVA) following Bonferroni *post hoc* test using Prism Graphpad 5 software. *P* < 0.05 was set for statistical significance.

## RESULTS

### Se-PFPs inhibit cell proliferation and induce apoptosis

Our recent study demonstrated that Se-PFPs significantly inhibited cell proliferation and induced cell apoptosis in MDA-MB-cells (data not shown). Here we examined the effects of Se-PFPs in OC cells. Se-PFPs significantly suppressed the proliferation of HEY and SKOV3 cells at 24 and 48 hrs in a concentration-dependent (between 100-1000 μg/ml) manner (*p* < 0.05, Figure 1A and 1B). Interestingly, different doses of Se-PFPs didn't show significantly inhibitory effect on the proliferation of HOSE cells, an immortalized non-tumorigenic human ovarian surface epithelial cell line (Supplementary Figure S1A). To clarify whether reduced cell proliferation after Se-PFPs treatment is caused by cell death, we carried out cell apoptosis assays using multiple methods. Annexin V and PI staining showed that treatment of 200 and 400 μg/ml Se-PFPs for 24 hrs caused cell apoptosis by 21.3% and 41.4% in HEY cells, and by 16.7% and 30.4% in SKOV3 cells, respectively (*P*<0.05, Figure 1C and Supplementary Figure S1B). The apoptosis induction was validated by elevated PARP, caspase-3 cleavage and Bax expression, and decreased Bcl-2 expression in Se-PFPs-treated HEY and SKOV3 cells (Figure 1D), but the mRNA level of Bcl-2 and Bax was not affected by Se-PFPs treatment in both cells (Supplementary Figure S1E). Moreover, 200 and 400 μg/ml Se-PFPs significantly increased the activities of caspase-3 and -9 (*P*<0.05, Supplementary Figure S1C and S1D). Additionally, compared with 200 μg/ml Se-PFPs, 400 μg/ml Se-PFPs exhibited significantly stronger effect on inducing cell apoptosis (*P<0.05*, Figure 1C and Supplementary Figure S1C and S1D).

**Figure 1:** Se-PFPs inhibit cell proliferation and induce cell apoptosis **A.** HEY cells and **B.** SKOV3 cells were incubated with indicated doses of Se-PFPs for 24 and 48 hrs, respectively. Cell viability was detected using MTT method. The data are presented as the ratio to the untreated cells. **C.** Se-PFPs induce cell apoptosis. The apoptotic cells were examined by Annexin V and PI staining and analyzed by flow cytometry. **D.** Se-PFPs affect the cleavage (PARP and caspase-3) and expression (Bcl-2 and Bax) of apoptosis-associated proteins. β-actin was used as a control. The statistical analysis was carried out by using one-way ANOVA following Bonferroni *post hoc* test, and different letters above each column represent statistical difference at a level of *p* < 0.05 (n=3).

### Se-PFPs inhibit epithelial-mesenchymal transition (EMT)

It has been demonstrated that both selenium and polysaccharides can inhibit EMT in primary cells and cancer cell lines [25, 26], suggesting that Se-PFPs could inhibit EMT in OC cells. Indeed, 200 and 400 μg/ml Se-PFPs treatment for 48 hrs significantly increased the expression (at mRNA and protein levels) of epithelial markers E-cadherin and cytokeratin 19, but significantly decreased the expression (at mRNA and protein levels) of mesenchymal markers including ZEB1, ZEB2, N-cadherin and vimentin in HEY and SKOV3 cells (*P<0.05*, Figure 2A and 2B). Moreover, 400 μg/ml Se-PFPs exhibited more significant effects on upregulating or downregulating mRNA expression of these genes compared with 200 μg/ml Se-PFPs (*P<0.05*, Figure 2A). Furthermore, 200 and 400 μg/ml Se-PFPs treatment showed similar effects on protein expression of EMT markers as seen on mRNA expression of these genes (*P<0.05*, Figure 2B). Thus, Se-PFPs inhibit EMT capacity in HEY and SKOV3 cells.

**Figure 2:** Se-PFPs treatment inhibits EMT change in HEY and SKOV3 cells HEY and SKOV3 cells were treated with 200 μg/ml and 400 μg/ml Se-PFPs for 48 hrs, the expression of E-Cadherin, Cytokeratin 19, N-Cadherin, vimentin, ZEB1 and ZEB2 was measured by real-time PCR **A.** and Western blot **B.** β-actin was used as a control. The statistical analysis was carried out by using one-way ANOVA following Bonferroni *post hoc* test, and different letters above each column represent statistical difference at a level of *p* < 0.05 (n=3).

### Se-PFPs inhibit cell migration and invasion

Since Se-PFPs inhibited EMT, we sought to examine the effects of Se-PFPs on cell migration and invasion. Transwell assay showed that 200 and 400 μg/ml Se-PFPs treatment significantly inhibited HEY and SKOV3 cell migration (*P<0.05*, Figure 3A). Inhibitory effect of Se-PFPs on cell migration was validated by wound healing assay (Figure 3B). In the meantime, Se-PFPs treatment significantly decreased the invasive capacity of HEY and SKOV3 cells (*P*<0.05, Figure 3C). MMP-9 is a key regulator for tumor migration and invasion [27]. Here we assessed the expression and activity of MMP-9 after Se-PFPs treatment. The protein expression (not mRNA) and activity of MMP-9 were significantly suppressed by Se-PFPs treatment in HEY and SKOV3 cells (*P*<0.05, Figure 3D and 3E, and Supplementary Figure S1E), indicating that MMP-9 may be involved in the anti-migratory and anti-invasive activities of Se-PFPs. Moreover, compared with 200 μg/ml Se-PFPs, 400 μg/ml Se-PFPs exhibited significantly stronger effect on inhibiting cell migration and invasion (*P<0.05*, Figure 3A–3E).

**Figure 3:** Se-PFPs inhibit cell migration and invasion in HEY and SKOV3 cells **A.** Effect of Se-PFPs on cell migration using transwell migration assay. **B.** Validation of cell migration using wound healing assay. Representative images were shown in the left (scale bar = 500 μm); while the statistical graph was presented in the right. **C.** Effect of Se-PFPs on cell invasion using Matrigel invasion assay. After 24 hrs, the migrated or invaded HEY and SKOV3 cells were fixed, stained, and counted under a microscope. Some representative images from HEY cells are exhibited (left). For the statistics (right), the data are presented as the ratio to the untreated cells, scale bar = 100 μm. **D.** Effect of Se-PFPs on MMP-9 expression in HEY and SKOV3 cells after 48 hrs. β-actin was used as a control. **E.** Effect of Se-PFPs on MMP-9 activity in cell culture supernatant. The statistical analysis was carried out by using one-way ANOVA following Bonferroni *post hoc* test, and different letters above each column represent statistical difference at a level of *p* < 0.05 (n=3).

### Antitumor activity of Se-PFPs *in vivo*

To verify whether our *in vitro* findings could be recapitulated *in vivo*, the antitumor activity of Se-PFPs was performed in HEY xenografted model. Nude mice were injected with HEY cells and simultaneously treated with 400 μg/ml Se-PFPs or equal volume of vehicle. The mice treated with Se-PFPs displayed decreased tumor volume after 21 days and reduced tumor weight compared with vehicle control mice (*P<0.05*, Figure 4A and 4B). However, there were no differences in body weight and adverse effects between the control and Se-PFPs-treated groups (data not shown). The immunohistochemical staining of Ki-67 and TUNEL revealed that the ratio of Ki-67 positive cells was significantly decreased while the ratio of TUNEL positive cells was significantly elevated in xenografted tumor tissues from Se-PFPs-treated mice (*P<0.05*, Figure 4C). Moreover, the expression of Bcl-2, N-cadherin, vimentin and MMP-9 were decreased, while the expression of Bax and E-cadherin was elevated in xenografted tumor tissues from Se-PFPs-treated mice (Figure 4D). Consistent with the findings of *in vitro* experiments, these results from *in vivo* experiments support the antitumor activity of Se-PFPs.

**Figure 4:** Antitumor activity of Se-PFPs in HEY-xenografted nude mice The volume **A.** and weight **B.** of tumors from HEY-xenografted nude mice were shown. HEY cells (1 × 10^6^) were injected subcutaneously into nude mice, and then administered with PBS or Se-PFPs (400 mg/day/kg weight) by gavage for 28 consecutive days. The tumor size was measured every 7 days. After 28 days of treatment, the mice were euthanized by CO2 inhalation. The tumors were separated and weighed. **C.** IHC staining for proliferation marker Ki-67 and TUNEL positivity, and scale bar represents 50 μm in Ki-67 staining and 500 μm in TUNEL staining, respectively. **D.** Western blot analysis was performed to determine the expression of Bax, Bcl-2, E-cadherin, N-cadherin, vimentin, MMP-9 and nuclear β-catenin in xenografted tumor tissues. β-actin was used as a control. **E.** IHC staining for nuclear β-catenin in tumors from HEY-xenografted nude mice. Scale bar = 50 μm. The statistic analysis was carried out by student's t-test. *P<0.05.

### Se-PFPs inhibit Wnt/β-catenin signaling pathway

The Wnt/β-catenin pathway is one of the major signaling pathways thought to be involved in EMT in OC (7). β-catenin is mainly localized in cytoplasm and nucleus, while nuclear accumulation of β-catenin indicates the activation of its oncogenic form, which can lead to cancer cell growth and poor prognosis (7). So we sought to test whether β-catenin is involved in the antitumor activity of Se-PFPs. Indeed, active nuclear β-catenin expression in the tumors from Se-PFPs-treated mice was also decreased obviously (Figures 4D and 4E). Moreover, Se-PFPs treatment significantly inhibited β-catenin expression particularly nuclear β-catenin expression in HEY and SKOV3 cells, which effect was dose- and time-dependent (Figure 5A and Supplementary Figure S2A). We further examined the effect of Se-PFPs on cyclin D1, a direct target of Wnt/β-catenin pathway. 400 μg/ml Se-PFPs treatment significantly inhibited cyclin D1 expression in both HEY and SKOV3 cells (Figure 5A). To explore whether the downregulation of β-catenin in Se-PFPs-treated cells is caused by reduced protein synthesis or increased protein degradation, HEY and SKOV3 cells were treated with 400 μg/ml Se-PFPs and/or 20 μg/ml cycloheximide (CHX), an inhibitor of protein synthesis. β-catenin expression was not affected by Se-PFPs and/or cycloheximide treatment for 30 min (Supplementary Figure S2B), however, after 24 h treatment, β-catenin expression in HEY and SKOV3 cells was obviously downregulated by CHX, dramatically reduced by Se-PFPs and completely blocked by the combination of CHX and Se-PFPs (Figure 5B). These data indicate that the downregulation of β-catenin in Se-PFPs-treated cells may be caused by increased degradation.

**Figure 5:** Se-PFPs suppress β-catenin signaling in a GSK-3β–dependent mechanism **A.** Se-PFPs inhibit the expression of cytoplasmic and nuclear β-catenin and cyclin D1 in HEY and SKOV3 cells. HEY and SKOV3 cells were incubated with the indicated doses of Se-PFPs for 48 hrs. α-tubulin was used as a loading control for cytoplasmic proteins, while lamin A/C was an internal control for nuclear proteins. **B.** Protein synthesis inhibitor, cycloheximide (CHX), reduces β-catenin expression in Se-PFPs-treated HEY and SKOV3 cells. The cells were incubated with 20 μg/ml of CHX in the presence or absence of Se-PFPs (400 μg/ml) for 24 hrs. **C.** Se-PFPs inhibit GSK-3β phosphorylation, leading to elevated phosphorylation of β-catenin in HEY and SKOV3 cells. HEY and SKOV3 cells were incubated with the indicated doses of Se-PFPs for 48 hrs. **D.** GSK-3β inhibitor, LiCl, increases GSK-3β phosphorylation and thus inhibits β-catenin phosphorylation in HEY and SKOV3 cells. The cells were treated with indicated concentrations of LiCl for 2 hrs. **E.** LiCl completely neutralizes the inhibitory effect of Se-PFPs on β-catenin expression. HEY and SKOV3 cells were treated with different doses of LiCl for 2 hrs in the presence of 400 μg/ml Se-PFPs. **F.** Proteasome inhibitor MG132 can rescue β-catenin expression in Se-PFPs-treated HEY and SKOV3 cells. HEY and SKOV3 cells were treated with Se-PFPs for 18 hrs, and co-treated with 5 μM MG132 for another 6 hrs. β-actin was used as a loading control.

It is well-established that GSK-3β is a key regulator for β-catenin degradation in Wnt/β-catenin pathway (7), we sought to examine the expression of total GSK-3β and phosphorylated GSK-3β in HEY and SKOV3 cells after Se-PFPs treatment. Se-PFPs treatment didn't affect the expression of total GSK-3β, while the level of phosphorylated GSK-3β was significantly decreased in HEY and SKOV3 cells after Se-PFPs treatment (Figure 5C). Moreover, the level of phosphorylated β-catenin in HEY and SKOV3 cells was elevated after Se-PFPs treatment (Figure 5C). To further verify GSK-3β is involved in the phosphorylation of β-catenin in Se-PFPs-treated cells, HEY and SKOV3 cells were treated with 400 μg/ml Se-PFPs and/or different concentrations of lithium chloride (LiCl), a specific inhibitor of GSK-3β. LiCl treatment only increased the level of phosphorylated GSK-3β in a concentration-dependent manner in both cell lines, indicating the inhibition of GSK-3β (Figure 5D). By contrast, the level of phosphorylated β-catenin was significantly decreased after LiCl treatment in a concentration-dependent manner although the level of total β-catenin was not obviously changed (Figure 5D). Furthermore, in the presence of various doses of LiCl, Se-PFPs treatment didn't change β-catenin expression in HEY and SKOV3 cells (Figure 5E). Besides GSK-3β inhibitor, we also observed a proteasome inhibitor MG132 could completely restore β-catenin expression in Se-PFPs-treated HEY and SKOV3 cells (Figure 5F).

### Se-PFPs inhibit cell growth and invasive potential via inhibiting β-catenin signaling

To verify β-catenin is involved in the inhibition of cell proliferation and invasion in Se-PFPs-treated cells, we stably inhibited β-catenin expression at mRNA and protein levels using two different shRNAs or overexpressed β-catenin in HEY and SKOV3 cells (*P<0.05*, Figure 6A and 6B). Moreover, overexpression of LV-β-catenin in Se-PFPs-treated HEY and SKOV3 cells could rescue the protein expression of β-catenin to the level similar to untreated control cells (Figure 6B). We further examined the effects of β-catenin (knockdown and overexpression) on the expression of Bcl-2, Bax, MMP-9, E-cadherin, N-cadherin and Vimentin, which are upregulated or downregulated by Se-PFPs treatment. Similar to Se-PFPs treatment, β-catenin knockdown by two shRNAs significantly decreased the expression of Bcl-2, MMP-9, N-cadherin and Vimentin and significantly increased the expression of Bax and E-cadherin in HEY and SKOV3 cells (Figure 6C), while β-catenin overexpression exerted the opposite effects on the expression of these proteins (Figure 6D). These results support β-catenin is involved in the changes in cell apoptosis, inhibition of EMT and invasion after Se-PFPs treatment. Next we predicted that β-catenin knockdown in OC cells could induce similar effects on cell proliferation and invasion as seen in Se-PFPs-treated cells, and exogenous β-catenin could neutralize the effects of Se-PFPs on cell proliferation and invasion. Indeed, depletion of β-catenin in HEY and SKOV3 cells significantly inhibited cell viability and invasive potential, which was comparable to Se-PFPs treatment (Figures 7A and 7C). By contrast, β-catenin overexpression in HEY and SKOV3 cells significantly increased cell viability and invasive potential, particularly neutralized the inhibitory effects of Se-PFPs on cell proliferation and invasion (Figures 7B and 7D). Additionally, empty vector and negative control shRNA didn't change cell viability and invasion in HEY and SKOV3 cells (Figure 7B–7D). Hence, the antitumor activity of Se-PFPs in OC cells is achieved by inhibition of β-catenin signaling.

**Figure 6:** β-catenin signaling regulates the expression of apoptosis- and EMT-related genes HEY and SKOV3 cells were treated with 400 μg/ml Se-PFPs, or infected with lentivirus particles carrying empty vector, β-catenin, negative control shRNA (NC shRNA), β-catenin shRNA1 or β-catenin shRNA2 for 8 hrs, or left untreated. 48 hrs after infection, β-catenin mRNA expression was determined by real-time PCR **A.** and protein level was determined by Western blot **B. C.** Effect of β-catenin knockdown on the expression of Bcl-2, Bax, MMP-9, E-cadherin, N-cadherin and Vimentin. **D.** Effect of β-catenin overexpression on the expression of Bcl-2, Bax, MMP-9, E-cadherin, N-cadherin and Vimentin. β-actin was used as a loading control.

**Figure 7:** β-catenin signaling is involved in the antitumor activity of Se-PFPs **A.** β-catenin knockdown inhibits cell viability in HEY and SKOV3 cells. **B.** β-catenin overexpression increases cell viability in HEY and SKOV3 cells and rescues cell viability in Se-PFPs-treated HEY and SKOV3 cells. MTT was used to detect the cell viability. The cell viability of control group was set at 100%, and the data of experimental groups were presented as the ratio to the control group. **C.** β-catenin knockdown decreases cell invasion in HEY and SKOV3 cells. **D.** β-catenin overexpression promotes cell invasion in HEY and SKOV3 cells and rescues cell invasion in Se-PFPs-treated HEY and SKOV3 cells. The invasive potential of HEY and SKOV3 cells was assessed. The statistical analysis was carried out by using one-way ANOVA following Bonferroni *post hoc* test, and different letters above each column represent statistical difference at a level of *p* < 0.05 (n=3).

## DISCUSSION

The antitumor activity of polysaccharides from various medicinal plants has been demonstrated in ovarian cancer cells, which is mostly associated with the inhibition of cell proliferation, migration and invasion, and the induction of cell apoptosis [28, 29]. Se has also been found to play a role in prevention and treatment of ovarian cancer [30, 31]. In the body, inorganic Se can be transformed into organic Se by coupling with polysaccharides or proteins, which makes it less toxic or much safer. Hence, it is reasonable to predict that Se-enriched polysaccharides may have significant antitumor effect. Recent studies reported the antitumor/antiproliferative activity of Se-enriched polysaccharides in human osteosarcoma [22], breast cancer [19] and multiple cancer cell lines [23]. Moreover, we successfully purified Se-enriched polysaccharides from *P. Fortuneana* (Se-PFPs) [21] and also found the antiproliferative activity of Se-PFPs in human breast cancer cell line MDA-MB-231 (data not shown). This evidence suggests that Se-PFPs may have antitumor activity in other cancers.

Polysaccharides exert antitumor activity through various signaling pathways such as NF-kB [32], PI3K/AKT [33], and MAPK [34]. In the present study, we firmly demonstrated the antitumor activity of Se-PFPs in OC using *in vitro* and *in vivo* experiments. More importantly, our detailed mechanistic insights indicate that the antitumor activity of Se-PFPs in OC is achieved by the inhibition of Wnt/β-catenin signaling pathway. These results are supported by previous findings: 1) polysaccharides can suppress tumor growth, invasion, and angiogenesis through the inhibition of Wnt/β-catenin signaling in colon cancer cells [35]; 2) Se is a key regulator of the Nrf2 and Wnt signaling pathways, in which Se deficiency leads to the activation of Nrf2 and Wnt pathways [36]. In cells, β-catenin plays two major roles: forming adherens junction with E-cadherin and acting as a transcriptional factor to regulate target genes expression [7]. β-catenin plays a dominant role in cancer progression through mediating cell cycle transition and cell apoptosis [7, 37]. Cyclin D1 is a key inducer of transition from the G1 to S phase of cell cycle and is directly regulated by β-catenin-TCF (T-cell factor) complex [38]. Consistently, Se-PFPs treatment dramatically inhibited the expression of β-catenin (particularly nuclear β-catenin) and cyclin D1, and thus led to the inhibition of cell proliferation in HEY and SKOV3 cell lines and HEY-xenografted tumors. By contrast, β-catenin signaling can inhibit cell apoptosis through mediating Bcl-2 activity or inhibiting Bax expression [39, 40]. Moreover, polysaccharides can induce caspase-dependent cell apoptosis [41, 42], and the antitumor activity of Se is mostly gained by the inhibition of cell cycle/proliferation and induction of cell apoptosis [43]. It is commonly accepted that anti-cancer agents regulate functions of the multidomain Bcl-2 family members (such as to activate Bax or to neutralize Bcl-2) via modulating the expression of short half-life proteins (e.g., BH3-only). This evidence strongly support our findings that Se-PFPs treatment significantly induced cell apoptosis in *in vitro* cell lines and *in vivo* xenografted tumors, accompanied by elevated BAX expression, PARP and caspase-3 cleavage and activities of caspase-3 and caspase-9, and decreased level of Bcl-2.

β-catenin is closely associated with the migration and invasion of ovarian cancer cells, these functions are mostly achieved by inducing EMT change and enhancing the activity of MMP-2 and MMP-9 [44–46]. Moreover, polysaccharides have been found to suppress cancer cell migration and invasion through the inhibition of EMT and MMPs activity [26, 47]. Although the inhibitory effects of Se on cell migration and invasion have been rarely studied, here we firmly demonstrated Se-PFPs are a strong suppressor for cell migration and invasion in HEY and SKOV3 cells. This conclusion is drawn mostly based on reduced MMP-9 activity and EMT inhibition (elevated epithelial markers such as cytokeratin 19 and E-cadherin and reduced mesenchymal markers such as vimentin, N-cadherin, ZEB1 and ZEB2) in Se-PFPs-treated cells. More importantly, our results demonstrated that β-catenin ablation in HEY and SKOV3 cells exerted similar effects as Se-PFPs treatment on cell viability and invasion. Conversely, β-catenin overexpression can completely neutralize the inhibitory effects of Se-PFPs on cell viability and invasion. Hence, it is reasonable to conclude that the inhibitory effects of Se-PFPs on cell proliferation, migration and invasion are achieved by the inhibition of β-catenin signaling.

Since the inhibitory effect of polysaccharides on β-catenin signaling in cancer cells is rarely reported, the mechanistic insights for this regulation remain elusive. However, Se has been reported as a key negative regulator for Wnt/β-catenin signaling pathways [36]. Under unstimulated or inhibitory state of classic canonical β-catenin pathway, β-catenin in the cytosol closely associates with a “degradation complex” including adenomatous polyposis coli (APC), Axin and GSK-3β and casein kinase-1 (CK1), and is phosphorylated by GSK-3β and degraded by ubiquitin-proteasome pathway (UPP), which results in low level of nuclear β-catenin[7, 47]. By contrast, upon binding with Wnt proteins, Wnt receptors Frizzleds will recruit Axin to the membrane via the adapter protein disheveled (Dvl) and cause the phosphorylation and degradation of GSK-3β due to the destruction of “degradation complex”, and thus results in release and nuclear translocation of β-catenin [7, 48]. Our results strongly support that the inhibitory effect of Se-PFPs on β-catenin signaling is GSK-3β-dependent in HEY and SKOV3 cells, because Se-PFPs treatment markedly decreased the level of phosphorylated GSK-3β and the inhibition of GSK-3β by LiCl could block the inhibitory effect of Se-PFPs on β-catenin expression. Moreover, Se-PFPs treatment caused obvious decrease in cytoplamic β-catenin level and remarkable decrease in nuclear β-catenin level, while phosphorylated β-catenin level was dramatically elevated upon Se-PFPs treatment. Because phosphorylated β-catenin is degraded by UPP, this is the main reason for decreased cytoplamic and nuclear β-catenin in Se-PFPs-treated cells. This reason is also supported by the evidence that the inhibition of proteasome by MG132 completely rescued the inhibitory effect of Se-PFPs on β-catenin expression. Furthermore, protein synthesis inhibitor CHX further reduced β-catenin expression in Se-PFPs-treated cells. These findings strongly support that the inhibitory effect of Se-PFPs on β-catenin expression is caused by GSK-3β-dependent β-catenin degradation.

In summary, Se-PFPs exert antitumor effect on OC cells through inhibiting cell proliferation, migration, invasion and EMT, and inducing cell apoptosis. These effects are achieved by the inhibition of β-catenin signaling. Thus Se-PFPs can be used as a potential preventative or therapeutic agent for OC patients.

## SUPPLEMENTARY MATERIALS FIGURES AND TABLE



## Abbreviations

Se-PFPs: selenium-enriched *Pyracantha fortuneana* (Maxim.) Li polysaccharides
MTT: 3-(4,5-Dimethylthiazol-2-yl)-2,5-diphenyltetrazolium bromide
DMSO: dimethyl sulfoxide
BSA: bovine serum albumin
PI: propidium iodide
PARP: poly (ADP-ribose) polymerase
DMEM: dulbecco modified eagle medium
DAPI: 4′,6-diamidino-2-phenylindole
b.w.: body weight
RIPA: radio-immuno precipitation assay
MMP: matrix metalloproteinase
EMT: epithelial-mesenchymal transition
MET: mesenchymal-epithelial transition
HPLC: high performance liquid chromatography
TUNEL: TdT-mediated dUTP nick end labeling
